The article "Outcomes of Direct-Acting Antivirals Versus Interferon-Based Therapy in Chronic Hepatitis C Infection" was retracted in 2025. Reasons: unreliable results or conclusions; concerns about the authorship.

# Outcomes of Direct-Acting Antivirals Versus Interferon-Based Therapy in Chronic Hepatitis C Infection

**DOI:** 10.7759/cureus.75902

**Published:** 2024-12-17

**Authors:** Ratna Chowdhury, Wardah Rashid, Taranpreet Singh, Abdur Rehman, Nida F Daterdiwala, Varaidzo Mkosi, Bhumikala Limbu, Syeda Alliza Bukhari, Afif Ramadhan, Muath M Dabas, Abdullah Shehryar, Ramadan Khan

**Affiliations:** 1 Internal Medicine, Saint James School of Medicine, Arnos Vale, VCT; 2 Internal Medicine, Khawaja Muhammad Safdar Medical College, Sialkot, PAK; 3 Internal Medicine, Mahatma Gandhi Mission (MGM) Medical College and Hospital, Mumbai, IND; 4 Surgery, Mayo Hospital, Lahore, PAK; 5 Internal Medicine, Ziauddin University, Karachi, PAK; 6 Internal Medicine, Ternopil National Medical University, Ternopil, UKR; 7 Emergency Medicine, Bishweshwar Prasad Koirala Institute of Health Sciences, Dharan, NPL; 8 Internal Medicine, Jinnah Sindh Medical University, Karachi, PAK; 9 Internal Medicine, Universitas Gadjah Mada, Yogyakarta, IDN; 10 General Surgery, University of Jordan, Amman, JOR; 11 Internal Medicine, Allama Iqbal Medical College, Lahore, PAK; 12 Internal Medicine, Dera Ghazi Khan Medical College, Dera Ghazi Khan, PAK

**Keywords:** antiviral efficacy, chronic hepatitis c, cirrhosis, direct-acting antivirals (daas), hcv treatment outcomes, hepatitis c genotypes, interferon-based therapy, pegylated interferon, ribavirin, sustained virologic response (svr)

## Abstract

This systematic review evaluates the outcomes of direct-acting antivirals (DAAs) compared to interferon-based therapies in patients with chronic hepatitis C infection. DAAs consistently demonstrate higher sustained virologic response (SVR) rates and better safety profiles across various patient populations, including those with cirrhosis and treatment-experienced individuals. The studies included highlight the superior efficacy of DAAs, with fewer adverse events such as anemia and fatigue, making them more tolerable and suitable for long-term treatment. These findings reinforce the clinical importance of DAAs as the standard of care for managing hepatitis C virus (HCV), particularly in special populations. Although interferon-based therapies remain relevant in resource-limited settings, this review emphasizes the need for broader access to DAAs to improve global health outcomes and reduce HCV-related morbidity and mortality.

## Introduction and background

Chronic hepatitis C virus (HCV) infection remains a significant global public health challenge, affecting an estimated 50 million people worldwide. The disease is a major cause of liver-related morbidity and mortality, often progressing to complications such as cirrhosis, hepatocellular carcinoma, and liver failure [1]. Traditionally, the mainstay of treatment for chronic hepatitis C involved interferon-based regimens, which combined pegylated interferon and ribavirin. However, these treatments were plagued by suboptimal cure rates, lengthy treatment durations, and significant adverse effects, making patient compliance a considerable issue [2].

The article "Outcomes of Direct-Acting Antivirals Versus Interferon-Based Therapy in Chronic Hepatitis C Infection" was retracted in 2025. Reasons: unreliable results or conclusions; concerns about the authorship.

The advent of direct-acting antivirals (DAAs) has revolutionized HCV treatment, providing a shorter, more effective, and well-tolerated alternative. DAAs target specific viral proteins necessary for HCV replication, offering cure rates of over 95% in many patient populations [3]. As a result, interferon-free regimens have become the standard of care for HCV, although interferon-based treatments are still occasionally used in resource-limited settings [4]. Comparing the outcomes of DAAs with interferon-based therapies is essential to solidify DAAs' position as the superior treatment option for chronic HCV infection and to guide clinical decision-making, particularly in special populations such as cirrhotic or treatment-experienced patients [5].

The systematic review is structured using the PICO framework, ensuring a focused and organized approach to analyzing the available clinical evidence [6]. The population (P) targeted in this review includes patients with chronic hepatitis C infection, encompassing both treatment-naive and treatment-experienced individuals. The scope extends across various genotypes of the virus, with special consideration for populations such as those with cirrhosis. The intervention (I) under examination is the use of DAAs, including combinations of drugs like sofosbuvir, daclatasvir, simeprevir, and other widely prescribed DAAs. For comparison (C), interferon-based therapies are evaluated, specifically regimens involving pegylated interferon and ribavirin, with or without the addition of telaprevir or boceprevir. The key outcomes (O) analyzed in this review include sustained virologic response (SVR), the occurrence of adverse events, treatment discontinuation rates, and instances of virologic relapse. This PICO framework will guide the systematic selection and evaluation of studies, ensuring a thorough comparison of the efficacy and safety of DAAs versus interferon-based therapies in the treatment of chronic hepatitis C.

The primary objective of this systematic review is to compare the clinical outcomes of DAAs with interferon-based therapies in the treatment of chronic hepatitis C infection. This review aims to evaluate the efficacy of both treatment modalities in achieving SVR and to assess the safety profiles of DAAs compared to interferon-based therapies. By synthesizing data from randomized controlled trials and large-scale clinical studies, the review seeks to provide evidence-based recommendations for the preferred treatment approach, focusing on the impact of DAAs in diverse patient populations, including cirrhotic and treatment-experienced individuals. Ultimately, the findings will inform clinical practice and contribute to optimizing therapeutic strategies for chronic HCV infection.

The article "Outcomes of Direct-Acting Antivirals Versus Interferon-Based Therapy in Chronic Hepatitis C Infection" was retracted in 2025. Reasons: unreliable results or conclusions; concerns about the authorship.

## Review

Materials and methods

Search Strategy

Our search strategy was rigorously developed in accordance with the Preferred Reporting Items for Systematic Reviews and Meta-Analysis (PRISMA) guidelines [7] to identify studies comparing the outcomes of DAAs versus interferon-based therapies in patients with chronic hepatitis C infection. To ensure a comprehensive and systematic search, we utilized key electronic databases, including PubMed, Medline, Embase, the Cochrane Library, and Scopus. The search covered the inception of each database through October 2024, capturing all relevant studies published to date.

We employed a combination of keywords and Medical Subject Headings (MeSH) terms related to the topic of interest, including "chronic hepatitis C", "direct-acting antivirals", "interferon-based therapy", "sustained virologic response", and "randomized controlled trials". Boolean operators ('AND', 'OR') were used to refine the search for maximum relevance. Example search strings included: "direct-acting antivirals AND interferon-based therapy AND hepatitis C", "sustained virologic response AND DAAs AND interferon", and "HCV infection AND DAAs OR interferon-based treatment". To capture all relevant studies, we also reviewed the reference lists of all selected articles and searched clinical trial registries and relevant conference proceedings to identify unpublished or ongoing research.

We restricted our search to studies published in English, focusing on randomized controlled trials, meta-analyses, and systematic reviews. The inclusion criteria specifically targeted clinical trials comparing DAAs with interferon-based therapies, emphasizing SVR and safety profiles in patients with chronic hepatitis C infection.

Eligibility Criteria

The eligibility criteria for this systematic review were carefully defined to ensure the inclusion of studies directly relevant to the comparison of DAAs and interferon-based therapies in the treatment of chronic hepatitis C infection. We included only peer-reviewed research articles, focusing specifically on randomized controlled trials (RCTs) and clinical trials that assessed the efficacy and safety of these treatment modalities. The primary outcomes of interest were SVR, adverse events, treatment discontinuation rates, and virologic relapse in patients with chronic hepatitis C.

The article "Outcomes of Direct-Acting Antivirals Versus Interferon-Based Therapy in Chronic Hepatitis C Infection" was retracted in 2025. Reasons: unreliable results or conclusions; concerns about the authorship.

Studies were selected based on several key inclusion parameters: trials involving adult patients with chronic hepatitis C infection of any genotype, whether treatment-naive or treatment-experienced, were included. Only RCTs and clinical trials published in English, from the inception of each database to October 2024, were considered. Studies that compared DAAs (such as sofosbuvir, daclatasvir, and simeprevir) to interferon-based therapies (including pegylated interferon and ribavirin) were prioritized. Exclusion criteria included studies that were not RCTs or clinical trials, studies with insufficient outcome data, non-English studies, and those focusing on animal models or pediatric populations.

Data Extraction

The data extraction process for this systematic review was designed to ensure the accuracy and reliability of the collected data, focusing on comparing DAAs and interferon-based therapies in chronic hepatitis C patients. Two independent reviewers initially screened articles by title and abstract, classifying them as "relevant", "not relevant", or "possibly relevant". Full-text reviews were conducted for articles that passed the initial screening to confirm their eligibility. To maintain consistency, data were extracted using a standardized form in Microsoft Excel, which captured key information such as study design, population characteristics, interventions, outcomes (e.g., SVR, adverse events), and any limitations noted in the studies. Discrepancies between reviewers were resolved through discussion with a third reviewer, ensuring the integrity of the data extraction process. This structured approach ensured that all pertinent data were systematically gathered for comprehensive analysis in our review.

Data Analysis and Synthesis

Given the diversity of interventions and patient populations across the selected studies, we opted not to perform a meta-analysis. Instead, we focused on a qualitative synthesis of the findings from the clinical trials and randomized controlled trials comparing DAAs and interferon-based therapies in chronic hepatitis C treatment. This approach enabled a detailed examination of the efficacy and safety outcomes, such as SVR, adverse events, and treatment discontinuation rates, across different patient subgroups and treatment regimens.

The studies were categorized based on the treatment modality, patient characteristics (e.g., treatment-naive vs. treatment-experienced), and the presence of comorbidities like cirrhosis. This allowed for a comparative analysis of the effectiveness of DAAs versus interferon-based therapies. Through thematic synthesis, we identified common trends, such as the higher SVR rates and improved safety profiles associated with DAAs, as well as the challenges presented by interferon-based treatments, including higher rates of adverse events. Our narrative synthesis integrated these findings, providing a comprehensive overview of the comparative outcomes, discussing the clinical implications, and highlighting gaps in the current evidence to guide future research in the treatment of chronic hepatitis C.

The article "Outcomes of Direct-Acting Antivirals Versus Interferon-Based Therapy in Chronic Hepatitis C Infection" was retracted in 2025. Reasons: unreliable results or conclusions; concerns about the authorship.

Results

Study Selection Process

The study selection process began with a comprehensive search across five key databases - PubMed, Medline, Embase, Cochrane Library, and Scopus - identifying 252 records (Figure 1). After removing 39 duplicates, 213 records were screened for relevance, with 160 records excluded based on the inclusion criteria. Of the 53 reports sought for retrieval, 18 were not obtained, leaving 35 reports for full-text assessment. Ultimately, 25 reports were excluded due to reasons such as non-RCT design (10), focus on non-HCV populations (eight), and insufficient data on primary outcomes (seven), resulting in the inclusion of 10 studies for final qualitative analysis.

**Figure 1:** The PRISMA flowchart represents the study selection process. PRISMA: Preferred Reporting Items for Systematic Reviews and Meta-Analysis.

Characteristics of the Selected Studies

The selected studies for this systematic review included a wide range of patient populations with chronic hepatitis C, encompassing both treatment-naive and treatment-experienced individuals across various genotypes. Most trials compared the efficacy and safety of DAAs with interferon-based therapies. The outcomes of interest, primarily SVR, varied by patient genotype, treatment duration, and presence of cirrhosis, but DAAs consistently demonstrated higher SVR rates and better tolerability. Several studies also highlighted lower adverse event rates, particularly anemia and fatigue, with DAA regimens compared to interferon-based therapies, reinforcing DAAs as a more effective and safer treatment option. A summary of the characteristics of the included studies is given in Table 1.

**Table 1:** A summary of the characteristics of the key studies. HCV: Hepatitis C Virus; GT: Genotype; IL28B: Interleukin 28B (genetic variant associated with HCV treatment response); pegIFN: Pegylated Interferon; RBV: Ribavirin; eRVR: Extended Rapid Virologic Response; SVR12: Sustained Virologic Response 12 weeks post-treatment; DAAs: Direct-Acting Antivirals; EBR/GZR: Elbasvir/Grazoprevir; SOF/PR: Sofosbuvir/Peginterferon and Ribavirin; OBV/PTV/r: Ombitasvir/Paritaprevir/Ritonavir; DSV: Dasabuvir; METAVIR: Scoring system for liver fibrosis and cirrhosis; SVR24: Sustained Virologic Response 24 weeks post-treatment.

Study	Population (P)	Intervention (I)	Comparison (C)	Outcomes (O)	Study Design	Key Findings
Jacobson I et al. (2016) [8]	602 treatment-naive HCV genotype 1 patients (GT1b and GT1a), including a subset with compensated cirrhosis, stratified by IL28B genotype	Daclatasvir 60 mg daily + pegIFN/RBV for 24 weeks; additional 24 weeks of pegIFN/RBV for those without eRVR	Telaprevir 750 mg three times/day + pegIFN/RBV for 12 weeks, followed by 12 or 36 weeks of pegIFN/RBV depending on eRVR	SVR12: 85% for daclatasvir vs 81% for telaprevir in GT1b patients; anemia less common with daclatasvir (-29.1% difference); SVR12 associated with IL28B genotype and cirrhosis status	Phase 3, randomized, open-label, noninferiority study	Daclatasvir was noninferior to telaprevir + pegIFN/RBV for SVR12; lower rates of anemia and rash-related events with daclatasvir, supporting its use in combination with other DAAs
Lawitz E et al. (2013) [9]	826 previously untreated HCV patients: 327 with genotypes 1, 4, 5, or 6 (98% had GT1 or GT4); 499 with genotypes 2 or 3	Sofosbuvir + peginterferon alfa-2a + ribavirin for 12 weeks (GT1, 4, 5, 6); Sofosbuvir + ribavirin for 12 weeks (GT2, 3)	Peginterferon alfa-2a + ribavirin for 24 weeks (GT2, 3)	SVR12: 90% for sofosbuvir + pegIFN/RBV (GT1, 4, 5, 6); SVR12: 67% for both sofosbuvir + RBV and pegIFN/RBV (GT2, 3); fewer adverse events with sofosbuvir	Phase 3, randomized, open-label, noninferiority trial	Sofosbuvir + pegIFN/RBV achieved 90% SVR12 in GT1/4 patients; sofosbuvir + RBV noninferior to pegIFN/RBV in GT2/3 patients, with lower adverse events reported in the sofosbuvir group
Sperl J et al. (2016) [10]	257 patients with HCV genotype 1 or 4 infection, most were non-cirrhotic (83.1%) and treatment-naive (74.9%)	Elbasvir/Grazoprevir (50 mg/100 mg daily) for 12 weeks	Sofosbuvir (400 mg daily) + PegIFN/RBV for 12 weeks	SVR12: 99.2% for elbasvir/grazoprevir vs 90.5% for sofosbuvir + PegIFN/RBV; fewer safety events with EBR/GZR (0.8%) compared to SOF/PR (27.8%)	Phase 3, randomized, open-label trial	EBR/GZR demonstrated superior efficacy and safety, with significantly higher SVR12 and fewer adverse events compared to sofosbuvir + PegIFN/RBV
Osinusi A et al. (2013) [11]	60 treatment-naive HCV genotype 1 patients with unfavorable treatment characteristics (varied stages of liver fibrosis)	Sofosbuvir (400 mg daily) + weight-based ribavirin or low-dose ribavirin (600 mg daily) for 24 weeks	N/A (single-arm study with internal comparison between weight-based and low-dose ribavirin)	SVR24: 68% for weight-based ribavirin; 48% for low-dose ribavirin; common adverse events: headache, anemia, fatigue, nausea	Phase 2, randomized, open-label trial	SVR24 rates were higher with weight-based ribavirin (68%) compared to low-dose ribavirin (48%); the treatment regimen was generally well-tolerated, with no discontinuations due to adverse events
Poordad F et al. (2019) [12]	105 patients with HCV genotype 1a infection without cirrhosis	Ombitasvir/paritaprevir/ritonavir + dasabuvir (OBV/PTV/r + DSV) with low-dose ribavirin for 12 weeks	N/A (comparison to historic SVR12 rates for OBV/PTV/r + DSV with weight-based ribavirin)	SVR12: 89.5% overall, 94.9% excluding non-virologic failures; 1 patient had a significant hemoglobin drop (<10 g/dL); common adverse events were mild	Phase 3, open-label, multicenter trial	OBV/PTV/r + DSV with low-dose ribavirin showed good efficacy (89.5% SVR12), but did not meet noninferiority compared to weight-based ribavirin; tolerability was improved with low-dose ribavirin
Pott-Junior H et al. (2019) [13]	127 noncirrhotic patients with HCV genotype 1, including treatment-naive and those unresponsive to pegylated interferon and ribavirin	Sofosbuvir (400 mg daily) + Daclatasvir (60 mg daily) for 12 weeks; Sofosbuvir (400 mg daily) + Simeprevir (150 mg daily) for 12 weeks	N/A (two DAA regimens compared)	SVR12: 100% for sofosbuvir + daclatasvir; 93.3% for sofosbuvir + simeprevir; common adverse events: fatigue, headache, mood swings	Phase 3, randomized, open-label, noninferiority trial	Sofosbuvir + daclatasvir achieved higher SVR12 rates compared to sofosbuvir + simeprevir (100% vs 93.3%); noninferiority of SOF + SMV to SOF + DCV was not established
Pearlman BL et al. (2015) [14]	82 patients with HCV genotype 1a and Child's grade A cirrhosis; 61% null responders, 39% therapy-naive; 48% African American	Simeprevir (150 mg/day) + Sofosbuvir (400 mg/day) for 12 weeks	Peginterferon alfa 2b (1.5 mcg/kg/wk) + Ribavirin (1000-1200 mg/day) + Sofosbuvir (400 mg/day) for 12 weeks	SVR12: 93% with simeprevir + sofosbuvir vs 75% with peginterferon + ribavirin + sofosbuvir; lower relapse rate and better quality of life in the simeprevir + sofosbuvir group	Prospective, randomized, open-label trial	Simeprevir + sofosbuvir had significantly higher SVR12, better tolerability, and lower relapse rates compared to the interferon-containing regimen
Lawitz E et al. (2014) [15]	168 HCV genotype 1 patients; previous non-responders to peginterferon and ribavirin or treatment-naive; METAVIR F0-F2 (cohort 1) and F3-F4 (cohort 2)	Simeprevir (150 mg/day) + Sofosbuvir (400 mg/day) for 12 or 24 weeks, with or without ribavirin	N/A (comparison between DAA regimens)	SVR12: 92% overall; 90% in cohort 1, 94% in cohort 2; common adverse events: fatigue, headache, nausea	Phase 2, randomized, open-label trial	Simeprevir + sofosbuvir was highly effective and well tolerated in both treatment-naive and non-responder patients, with SVR12 rates of 92%; serious adverse events were rare (2%)
Asselah T et al. (2016) [16]	120 patients with HCV genotype 4 and compensated cirrhosis; treatment-naive or treatment-experienced	Ombitasvir (25 mg), Paritaprevir (150 mg), and Ritonavir (100 mg) + Ribavirin (weight-based) for 12 or 16 weeks	N/A (two treatment durations compared)	SVR12: 97% in the 12-week group, 98% in the 16-week group; common adverse events: asthenia, fatigue, headache, anemia	Phase 3, randomized, open-label, multicenter trial	Extending treatment to 16 weeks provided no additional benefit over 12 weeks in achieving SVR12 in HCV genotype 4 patients with cirrhosis; 12 weeks of treatment was highly effective and well tolerated
Kowdley KV et al. (2013) [17]	316 treatment-naive, non-cirrhotic HCV patients (genotypes 1, 4, 6); 11 with genotype 4, 5 with genotype 6	Sofosbuvir (400 mg) + Peginterferon + Ribavirin for 12 or 24 weeks	N/A (comparison between treatment durations)	SVR24: 89% in cohort A (12 weeks), 89% in cohort B (24 weeks), 87% in cohort C (12 weeks + sofosbuvir monotherapy or sofosbuvir + ribavirin); common adverse events: anemia, neutropenia	Phase 2, randomized, open-label, multicenter trial	Sofosbuvir-based regimens achieved high SVR24 rates, with no additional benefit from extending treatment beyond 12 weeks; well-tolerated with anemia and neutropenia primarily linked to Peginterferon and Ribavirin

The risk of bias was assessed across all selected studies to evaluate the validity and reliability of their findings. Most studies demonstrated a low risk of bias across key domains, including randomization processes, measurement of outcomes, and adherence to intended interventions. While a few studies had minor concerns, such as a lack of explicit randomization details or potential bias from open-label designs, these did not significantly impact the overall integrity of the data. The following table summarizes the risk of bias assessments for each study, providing a comprehensive overview of the methodological rigor in each trial (Table 2).

The article "Outcomes of Direct-Acting Antivirals Versus Interferon-Based Therapy in Chronic Hepatitis C Infection" was retracted in 2025. Reasons: unreliable results or conclusions; concerns about the authorship.

**Table 2:** Assessment of risk of bias across randomized studies on HCV treatment outcomes. SVR12: Sustained Virologic Response 12 weeks post-treatment; HCV: Hepatitis C virus.

Study	Randomization Process	Deviations from Intended Intervention	Missing Outcome Data	Measurement of Outcome	Selective Reporting	Overall Risk of Bias
Jacobson I et al. (2016) [8]	Low risk: Randomization was stratified	Low risk: Open-label, but interventions likely adhered to	Low risk: Data were complete for the majority of participants	Low risk: SVR12 outcomes were clearly defined	Low risk: All predefined outcomes reported	Low
Lawitz E et al. (2013) [9]	Low risk: Randomized design	Low risk: Open-label, but treatment adherence was likely high	Low risk: Missing data minimal and balanced between groups	Low risk: SVR12 outcomes measured reliably	Low risk: All outcomes clearly reported	Low
Sperl J et al. (2016) [10]	Low risk: Randomization clearly described	Low risk: No major deviations from intended interventions	Low risk: Minimal missing data, no significant bias	Low risk: Objective measures used for outcomes	Low risk: All relevant outcomes reported	Low
Osinusi A et al. (2013) [11]	Some concerns: Single-center, randomization details not explicit	Low risk: Adherence to intervention was monitored	Low risk: Data completeness was high	Low risk: Outcomes measured objectively	Low risk: All outcomes specified were reported	Low
Poordad F et al. (2019) [12]	Some concerns: Open-label, comparison to historic data introduces potential bias	Low risk: Adherence was likely good	Low risk: Minimal missing data	Low risk: Objective measures for SVR12 used	Low risk: Outcomes were fully reported	Low
Pott-Junior H et al. (2019) [13]	Low risk: Randomization method described	Low risk: No significant deviations from intended interventions	Low risk: Data completeness ensured	Low risk: Objective outcomes measured	Low risk: All relevant outcomes reported	Low
Pearlman BL et al. (2015) [14]	Low risk: Randomization process clearly defined	Low risk: No significant deviations reported	Low risk: Data completeness was adequate	Low risk: SVR12 outcomes measured consistently	Low risk: All predefined outcomes reported	Low
Lawitz E et al. (2014) [15]	Low risk: Randomization described well	Low risk: Interventions adhered to protocol	Low risk: Missing data handled appropriately	Low risk: Objective measurement of outcomes	Low risk: Outcomes reported as expected	Low
Asselah T et al. (2016) [16]	Low risk: Clear description of randomization	Low risk: No significant deviations from intended interventions	Low risk: Minimal missing data	Low risk: SVR12 outcomes measured appropriately	Low risk: Full reporting of all predefined outcomes	Low
Kowdley KV et al. (2013) [17]	Low risk: Well-described randomization process	Low risk: Adherence to interventions was good	Low risk: No major missing data	Low risk: Outcomes measured objectively	Low risk: No selective reporting detected	Low

Discussion

The findings from this systematic review underscore the superior efficacy of DAAs compared to interferon-based regimens across various patient populations. In trials like those by Jacobson I et al. [8] and Lawitz E et al. [9], DAAs demonstrated higher SVR rates, particularly in genotype 1 patients, with daclatasvir showing an 85% SVR12 compared to telaprevir’s 81%. Similarly, Lawitz E et al. [9] reported a remarkable 90% SVR12 with sofosbuvir plus peginterferon alfa-2a and ribavirin in patients with genotypes 1, 4, 5, and 6, compared to lower SVR rates in interferon-based treatments for genotypes 2 and 3. Notably, the safety profile of DAAs was consistently better, with fewer adverse events such as anemia and rash, making them more tolerable and improving patient compliance.

The article "Outcomes of Direct-Acting Antivirals Versus Interferon-Based Therapy in Chronic Hepatitis C Infection" was retracted in 2025. Reasons: unreliable results or conclusions; concerns about the authorship.

Furthermore, several studies highlighted the advantages of newer DAA combinations. Sperl et al. [10] demonstrated that elbasvir/grazoprevir achieved an SVR12 of 99.2%, significantly higher than sofosbuvir plus pegIFN/RBV (90.5%), with fewer adverse events. This pattern was consistent in Poordad F et al. [12] and Pott-Junior H et al. [13], where DAA-based regimens not only achieved superior virologic outcomes but also presented better safety profiles, particularly in non-cirrhotic and treatment-naive populations. These findings solidify the place of DAAs as the gold standard in chronic hepatitis C management, while also highlighting their efficacy in special populations, such as those with cirrhosis or previous treatment failure, aligning with or surpassing prior research in the field.

The findings of this systematic review are largely consistent with existing literature that highlights the superior efficacy and safety of DAAs compared to interferon-based therapies in treating chronic hepatitis C [18]. Numerous prior reviews have similarly reported higher SVR rates and fewer adverse events with DAAs [19]. Our review further reinforces these conclusions, showing comparable results in high-risk populations such as those with cirrhosis and treatment-experienced patients. For example, in studies like Asselah T et al. [16], SVR12 rates of 97-98% were achieved in cirrhotic patients treated with ombitasvir/paritaprevir/ritonavir plus ribavirin, consistent with findings from other trials included in this review. This alignment strengthens the argument that DAAs should be the standard of care, even in more challenging patient populations.

However, our review also identified some discrepancies and gaps when compared to previous studies. While most literature demonstrates excellent outcomes in cirrhotic patients, some studies in our review, such as Jacobson I et al. [8], highlighted variability in SVR rates depending on factors such as IL28B genotype and cirrhosis status, which are not universally emphasized in prior reviews. Additionally, while DAAs generally show a better safety profile, the incidence of adverse events such as anemia and fatigue remains underreported in certain populations, creating gaps in the full understanding of the safety landscape [20]. These findings suggest a need for more detailed subgroup analyses in future studies, particularly focusing on the long-term safety and efficacy of DAAs in diverse populations, including those with comorbidities and advanced liver disease.

The article "Outcomes of Direct-Acting Antivirals Versus Interferon-Based Therapy in Chronic Hepatitis C Infection" was retracted in 2025. Reasons: unreliable results or conclusions; concerns about the authorship.

The clinical implications of this systematic review are clear: DAAs should be prioritized as the standard of care for patients with chronic hepatitis C infection across all eligible populations [21]. The consistently higher SVR rates, coupled with significantly fewer adverse events, make DAAs not only more effective but also more tolerable compared to interferon-based therapies. This is particularly important for special populations, such as patients with advanced liver disease or those who have previously failed treatment [22]. Studies like Sperl J et al. [10] and Asselah T et al. [16] demonstrate that even in these higher-risk groups, DAAs maintain high efficacy and safety profiles, suggesting that clinicians should strongly consider DAA regimens, even for patients with cirrhosis or treatment experience. This review reinforces the notion that interferon-based therapies should be reserved only for situations where DAAs are unavailable, such as in certain resource-limited settings.

In clinical settings where both DAAs and interferon-based treatments are available, the decision to prioritize DAAs should be guided by their superior outcomes and patient compliance. Interferon-based regimens, while sometimes still used in resource-limited environments, are associated with higher rates of adverse events such as anemia, fatigue, and depression, making them less ideal, particularly in populations where treatment adherence is critical [23]. The availability of DAAs with shorter treatment durations, improved tolerability, and higher cure rates, as demonstrated in trials by Jacobson I et al. [8] and Poordad F et al. [12], underscores their utility in improving overall public health outcomes. In settings where DAAs may be cost-prohibitive, efforts should be made to secure access to these therapies through national and international health initiatives, ensuring that patients, especially those in low- and middle-income countries, receive optimal treatment.

One of the main limitations of this systematic review lies in the heterogeneity of the included studies, particularly with regard to variations in study design, patient populations, and treatment protocols. The studies reviewed encompassed a wide range of hepatitis C virus genotypes, disease stages, and treatment histories, which may introduce variability in the reported outcomes, such as SVR rates and adverse event profiles. Additionally, some studies had small sample sizes, particularly in special populations like cirrhotic or treatment-experienced patients, which could limit the statistical power to detect differences in these subgroups. Another limitation is the relatively limited data on certain genotypes (e.g., genotypes 5 and 6) and in resource-limited settings where interferon-based therapies may still be used. These factors may affect the generalizability of our conclusions to all patient populations and settings, highlighting the need for more large-scale, well-controlled trials in diverse and underrepresented populations to fully understand the efficacy and safety of DAAs.

The article "Outcomes of Direct-Acting Antivirals Versus Interferon-Based Therapy in Chronic Hepatitis C Infection" was retracted in 2025. Reasons: unreliable results or conclusions; concerns about the authorship.

Future research should focus on addressing the gaps identified in this review, particularly in underrepresented populations such as those with less common HCV genotypes (e.g., genotypes 5 and 6), and patients in resource-limited settings where interferon-based therapies are still used [24]. Large-scale trials are needed to evaluate the long-term efficacy and safety of DAAs in these populations, especially in those with comorbidities or advanced liver disease, where data remain limited. Additionally, as newer DAAs and combination therapies continue to emerge, future studies should prioritize head-to-head comparisons between different DAA regimens to identify the most effective and safest treatment protocols [25]. Furthermore, the development of shorter, more cost-effective DAA regimens should be explored, particularly for use in low- and middle-income countries, to improve accessibility and compliance. Emerging trends such as pan-genotypic DAAs and combination therapies targeting difficult-to-treat patient populations also warrant further investigation, as they hold the potential to further revolutionize hepatitis C treatment globally.

## Conclusions

This systematic review reinforces the clear superiority of DAAs over interferon-based therapies in treating chronic hepatitis C infection, demonstrating consistently higher SVR rates, fewer adverse events, and better patient compliance. The findings support integrating DAAs as the standard of care in clinical practice, especially in high-risk populations such as those with cirrhosis or previous treatment failures. While interferon-based therapies may still play a role in resource-limited settings, the overall efficacy, tolerability, and shorter treatment durations of DAAs make them the preferred choice. These results have significant implications for HCV treatment guidelines, suggesting that global efforts should be made to ensure access to DAAs, particularly in underserved regions, to improve patient outcomes and contribute to the eradication of HCV.

The article "Outcomes of Direct-Acting Antivirals Versus Interferon-Based Therapy in Chronic Hepatitis C Infection" was retracted in 2025. Reasons: unreliable results or conclusions; concerns about the authorship.

## References

[1] (2024). Hepatitis C. https://www.who.int/news-room/fact-sheets/detail/hepatitis-c.

[2] Palumbo E (2011). Pegylated interferon and ribavirin treatment for hepatitis C virus infection. Ther Adv Chronic Dis.

[3] Asselah T, Marcellin P, Schinazi RF (2018). Treatment of hepatitis C virus infection with direct-acting antiviral agents: 100% cure?. Liver Int.

[4] Solbach P, Wedemeyer H (2015). The new era of interferon-free treatment of chronic hepatitis C. Viszeralmedizin.

[5] Lynch EN, Russo FP (2023). Outcomes and follow-up after hepatitis C eradication with direct-acting antivirals. J Clin Med.

[6] Eriksen MB, Frandsen TF (2018). The impact of patient, intervention, comparison, outcome (PICO) as a search strategy tool on literature search quality: a systematic review. J Med Libr Assoc.

[7] Page MJ, McKenzie JE, Bossuyt PM (2021). The PRISMA 2020 statement: an updated guideline for reporting systematic reviews. BMJ.

[8] Jacobson I, Zeuzem S, Flisiak R (2016). Daclatasvir vs telaprevir plus peginterferon alfa/ribavirin for hepatitis C virus genotype 1. World J Gastroenterol.

[9] Lawitz E, Mangia A, Wyles D (2013). Sofosbuvir for previously untreated chronic hepatitis C infection. N Engl J Med.

[10] Sperl J, Horvath G, Halota W (2016). Efficacy and safety of elbasvir/grazoprevir and sofosbuvir/pegylated interferon/ribavirin: a phase III randomized controlled trial. J Hepatol.

[11] Osinusi A, Meissner EG, Lee YJ (2013). Sofosbuvir and ribavirin for hepatitis C genotype 1 in patients with unfavorable treatment characteristics: a randomized clinical trial. JAMA.

[12] Poordad F, Sedghi S, Pockros PJ (2019). Efficacy and safety of ombitasvir/paritaprevir/ritonavir and dasabuvir with low-dose ribavirin in patients with chronic hepatitis C virus genotype 1a infection without cirrhosis. J Viral Hepat.

[13] Pott-Junior H, Bricks G, Grandi G, Figueiredo SJ, Castelo FA (2019). Sofosbuvir in combination with daclatasvir or simeprevir for 12 weeks in noncirrhotic subjects chronically infected with hepatitis C virus genotype 1: a randomized clinical trial. Clin Microbiol Infect.

[14] Pearlman BL, Ehleben C, Perrys M (2015). The combination of simeprevir and sofosbuvir is more effective than that of peginterferon, ribavirin, and sofosbuvir for patients with hepatitis C-related Child's class A cirrhosis. Gastroenterology.

[15] Lawitz E, Sulkowski MS, Ghalib R (2014). Simeprevir plus sofosbuvir, with or without ribavirin, to treat chronic infection with hepatitis C virus genotype 1 in non-responders to pegylated interferon and ribavirin and treatment-naive patients: the COSMOS randomised study. Lancet.

The article "Outcomes of Direct-Acting Antivirals Versus Interferon-Based Therapy in Chronic Hepatitis C Infection" was retracted in 2025. Reasons: unreliable results or conclusions; concerns about the authorship.

[16] Asselah T, Hézode C, Qaqish RB (2016). Ombitasvir, paritaprevir, and ritonavir plus ribavirin in adults with hepatitis C virus genotype 4 infection and cirrhosis (AGATE-I): a multicentre, phase 3, randomised open-label trial. Lancet Gastroenterol Hepatol.

[17] Kowdley KV, Lawitz E, Crespo I (2013). Sofosbuvir with pegylated interferon alfa-2a and ribavirin for treatment-naive patients with hepatitis C genotype-1 infection (ATOMIC): an open-label, randomised, multicentre phase 2 trial. Lancet (London, England).

[18] Due OT, Chaikledkaew U, Genuino AJ, Sobhonslidsuk A, Thakkinstian A (2019). Systematic review with meta-analysis: efficacy and safety of direct-acting antivirals for chronic hepatitis C genotypes 5 and 6. Biomed Res Int.

[19] Majd Jabbari S, Maajani K, Merat S, Poustchi H, Sepanlou SG (2021). An updated systematic review and meta-analysis on efficacy of Sofosbuvir in treating hepatitis C-infected patients with advanced chronic kidney disease. PLoS One.

[20] Hayes KN, Burkard T, Weiler S, Tadrous M, Burden AM (2021). Global adverse events reported for direct-acting antiviral therapies for the treatment of hepatitis C: an analysis of the World Health Organization VigiBase. Eur J Gastroenterol Hepatol.

[21] Jakobsen JC, Nielsen EE, Feinberg J (2017). Direct-acting antivirals for chronic hepatitis C. Cochrane Database Syst Rev.

[22] Krassenburg LA, Zanjir WR, Georgie F, Stotland E, Janssen HL, Hansen BE, Feld JJ (2021). Evaluation of sustained virologic response as a relevant surrogate endpoint for long-term outcomes of hepatitis C virus infection. Clin Infect Dis.

[23] Seo KI, Yun BC, Li WJ, Lee SU, Han BH, Park ET (2017). Barriers to treatment of failed or interferon ineligible patients in the era of DAA: single center study. Clin Mol Hepatol.

[24] Umer M, Iqbal M (2016). Hepatitis C virus prevalence and genotype distribution in Pakistan: comprehensive review of recent data. World J Gastroenterol.

[25] Gupta V, Kumar A, Sharma P, Arora A (2017). Newer direct-acting antivirals for hepatitis C virus infection: perspectives for India. Indian J Med Res.

